RETRACTED

# Influences of Chronic Mild Stress Exposure on Motor, Non-Motor Impairments and Neurochemical Variables in Specific Brain Areas of MPTP/Probenecid Induced Neurotoxicity in Mice

**DOI:** 10.1371/journal.pone.0146671

**Published:** 2016-01-14

**Authors:** Udaiyappan Janakiraman, Thamilarasan Manivasagam, Arokiasamy Justin Thenmozhi, Musthafa Mohamed Essa, Rajamani Barathidasan, Chidambaram SaravanaBabu, Gilles J. Guillemin, Mohammed A. S. Khan

**Affiliations:** 1 Department of Biochemistry and Biotechnology, Annamalai University, Annamalainagar, 608002, Tamilnadu, India; 2 Department of Food Science and Nutrition, CAMS, Sultan Qaboos University, Muscat, Oman; 3 Ageing and Dementia Research Group, Sultan Qaboos University, Muscat, Oman; 4 Centre for Toxicology and Developmental Research, Sri Ramachandra University, Porur, Chennai-600 116, Tamilnadu, India; 5 Neuropharmacology group, Faculty of Medicine and Health Sciences, Deb Bailey MND Research Laboratory, Macquarie University, NSW, 2109, Australia; 6 Harvard Medical School, Massachusetts General Hospital, Shriners Hospital for Children, Boston, Massachusetts, 02114, United States of America; INSERM / CNRS, FRANCE

## Abstract

Parkinson's disease (PD) is regarded as a movement disorder mainly affecting the elderly population and occurs due to progressive loss of dopaminergic (DAergic) neurons in nigrostriatal pathway. Patients suffer from non-motor symptoms (NMS) such as depression, anxiety, fatigue and sleep disorders, which are not well focussed in PD research. Depression in PD is a predominant /complex symptom and its pathology lies exterior to the nigrostriatal system. The main aim of this study is to explore the causative or progressive effect of chronic mild stress (CMS), a paradigm developed as an animal model of depression in1-methyl-4-phenyl-1,2,3,6-tetrahydropyridine (25 mg/kg. body wt.) with probenecid (250 mg/kg, s.c.) (MPTP/p) induced mice model of PD. After ten i.p. injections (once in 3.5 days for 5 weeks) of MPTP/p or exposure to CMS for 4 weeks, the behavioural (motor and non-motor) impairments, levels and expressions of dopamine (DA), serotonin (5-HT), DAergic markers such as tyrosine hydroxylase (TH), dopamine transporter (DAT), vesicular monoamine transporters—2 (VMAT 2) and α-synuclein in nigrostriatal (striatum (ST) and substantia nigra (SN)) and extra-nigrostriatal (hippocampus, cortex and cerebellum) tissues were analysed. Significantly decreased DA and 5-HT levels, TH, DAT and VMAT 2 expressions and increased motor deficits, anhedonia-like behaviour and α-synuclein expression were found in MPTP/p treated mice. Pre and/or post exposure of CMS to MPTP/p mice further enhanced the MPTP/p induced DA and 5-HT depletion, behaviour abnormalities and protein expressions. Our results could strongly confirm that the exposure of stress after MPTP/p injections worsens the symptoms and neurochemicals status of PD.

RETRACTED

## Introduction

Parkinson’s disease (PD) is one of the most common, age related, neurodegenerative and movement disorders, arising mainly due to severe damage to the nigrostriatal pathway (resulting from the progressive loss of dopaminergic (DAergic) neurons in the substantianigra (SN) and the loss of dopamine (DA) terminals in the striatum (ST)) [1]. This leads to four cardinal motor symptoms including resting tremor, rigidity akinesia and postural instability (TRAP) in patients. Very recently only researchers have begun to focus on non- motor symptoms (NMS) of PD that are poorly recognised and inadequately treated by clinicians. In PD, mild lesions of the meso-limbic and meso-cortical pathways and involvement of non-dopaminergic systems (e.g.cholinergic, noradrenergic, serotoninergic) resulted in the appearance of non-motor symptoms such as anhedonia (reduced ability to experience pleasure), apathy, anxiety, panic attacks, social phobias and depression [2]. These non-motor symptoms precede the onset of motor symptoms and do not respond to the medication of the PD patients [3].

The exact cause of PD is still unknown. Swaab et al. [4] have concluded that stress abnormalities are progressive to various neurodegenerative diseases, including Alzheimer’s disease, Huntington’s disease and PD. Psychological stress is known to cause depression, anxiety and impaired cognition and are theorized to be one of the earliest proposed causes of PD. About 40–50% of all PD cases were reported to have depression [5] and it has been suggested that acute or chronic stress might lead to an earlier onset or worsen the motor symptoms of PD [6,7,8]. Moreover, stress along with corticosterone treatment exaggerated motor impairments and accelerated loss of midbrain dopamine producing neurons in 6-OHDA post-lesioned rats [9]. Recently Hemmerle et al. demonstrated that chronic stress-induced depression are concurrent, rather than preceding or following neurotoxin-induced neurodegeneration, which exacerbates the behavioural dysfunction and dopaminergic degeneration of nigrostriatal system [10].

Chronic Mild Stress (CMS) has been widely used in animals to imitate depressive disorders where the animals display similar patterns of stressful reactions like humans [11]. In the CMS paradigm, rodents are exposed to a variety of relatively mild stresses (e.g., isolated housing, disruption of light/dark cycles, and brief periods of food or water deprivation, tilting of home cages intermittently for relatively prolonged periods of time) that results in behavioural deficits and anhedonia, a core symptom of human depression [12]. Studies suggest that the pathology of depression in PD could lies outside the nigrostriatal pathway [13]. Several brain structures such as the hippocampus, cortex and cerebellum are known to have involvement in stress response and are reported to be affected by chronic exposure to stress [14,15,16].

RETRACTED

The present study is aimed to explore the causative, progressive or the combined effect of CMS in pre and/or post CMS exposed MPTP/p treated animals by evaluating motor dysfunctions and non-motor symptoms, the levels of dopamine, serotonin (5-HT) and the expressions of dopaminergic markers in the nigrostriatal (SN and striatum) and non-nigrostriatal (hippocampus, cortex and cerebellum) tissues.

## Materials and Methods

### Experimental procedures

#### Animals

Healthy adult Male C57BL/6 mice (25–30 g), purchased from the National Institute of Nutrition, Hyderabad, were housed in polypropylene cages with sterile paddy husk and maintained under ambient conditions of temperature and humidity. Food and water were provided ad libitum. All the experimental procedures pertaining to the use of the animals were in accordance with the guidelines of the Committee for the Purpose of Control and Supervision of Experiments on Animals (CPCSEA), New Delhi, India and approved by Annamalai University Animal Ethical Committee, Annamalai Nagar, Tamil Nadu, India (Reg No. 160/1999/CPCSEA) and the approval number: 893/2012.

Animals were allowed to acclimatise for 1 week prior to CMS exposure and MPTP/p dosing. During the acclimatisation period, mice were individually trained for the behaviour tasks.

#### Chemicals

MPTP, probenecid, anti-mouse TH and anti-mouse α-synuclein (Cell Signalling Technology, USA), anti-mouse DAT and anti-mouse VMAT-2 (Santa cruz, Biotechnology, USA) were used in this study. All other chemicals used were of analytical grade.

#### Grouping

Mice were randomly divided into six groups (n = 12). The Group I was saline treated control, Group II received MPTP/p (MPTP 25 mg/kg b.w in saline, s.c. and probenecid 250 mg/kg in 0.03 ml DMSO, i.p.) (5 weeks) [17], Group III was exposed to CMS (4 weeks). Group IV was exposed to pre-lesioned stress (MPTP/p followed by CMS), Group V was exposed to post lesioned stress (CMS followed by MPTP/p). Group VI was concomitant stress (2 week CMS before and after MPTP/p) (Fig 1).

**Fig 1:** Treatment schedule of the experimental study.

#### CMS Protocol

Mice were subjected to different kinds of stressors such as: cage tilting, damp sawdust, placement in an empty cage, grouped housing, placement in an empty cage with water on the bottom, placement of a foreign object in the cage, inversion of the light/dark cycle, food or water deprivation, lights on for a short period of time during the dark phase and switching cages [18]. On average, two of these stressors were applied daily at different times and following a semi-random 4-week schedule (Table 1).

RETRACTED

**Table 1:** The chronic mild stress protocol during the first week of the experiment. This schedule were followed for another three week.

Week 1	Sunday	Monday	Tuesday	Wednesday	Thursday	Friday	Saturday
Empty cage		10.00–13.00 h			9.30–12.30 h		15.00–17.00 h
Damp sawdust	9.00–12.00 h		9.00–12.00 h				
Cages tilt at 45°	14.00–17.00 h	14.00–17.00 h		10.00–13.00 h		9.00–10.30 h	
Water deprivation			17.00 h →	9.00 h			
Empty cage with water on the bottom				14.00–16.00 h			11.00–13.00 h
Continuous overnight illumination	17.00 h →	9.00 h			17.00 h →	9.00 h	
Food deprivation						17.00 h →	9.00 h
Light/dark succession every 15 min			23.00 h →	2.00 h			

### Behavioural assessment

#### Open field test

The apparatus (W100 cm×D100 cm×H40 cm) is made of wood and resin. The floor of this chamber was divided into 25 cm (5 × 5) squares. The mice were placed into one corner of an open field chamber and their behaviour was observed for 3 min. a). Number of squares explored; only when the animal enters a square with both its forelimb, one count is made. The number of centre squares (central 9 squares) and peripheral (the 16 squares adjacent to the wall) explored by the animal was noted separately. b). Number of grooming; i.e. consisting of licking the fur, washing face or scratching behaviour. c). Number of rearing; i.e. standing on hind limbs and sometimes leaning on the wall with forelegs, sniffing and looking around. The whole study was performed as blind study [19].

#### Narrow beam walking test

Animals were trained to walk on a narrow flat stationary wooden beam (L100 cm×W1 cm) placed at a height of 100 cm from the floor to reach an enclosed escape platform. The time taken to cross the beam from one end to the other and foot slip errors were also counted as described previously [19].

#### Sucrose Intake Test

Mice were exposed to two standard drinking bottles, containing 2.5% sucrose and the tap water, for every other night for 1 week. After this preliminary phase, mice were food deprived and exposed to the sucrose solution and water from 6:00 p.m. until 9.00 a.m. in the morning. The intake baseline for the sucrose solution was established, which corresponded to the average of three consecutive measurements. Once a week, mice were given a 15-h exposure to the sucrose solution and tap water in their home cage as described above. The position of the two bottles (right/left) was varied randomly from trial to trial. Sucrose intake was calculated as absolute intake (g) per group.

RETRACTED

At the end of the experiment (64^th^ day) after performing behavioural parameters, mice were anesthetized with an intraperitoneal injection of ketamine (75 mg/kg) and xylazine (5 mg/kg), and the brains of control and experimental mice were carefully removed, washed with 0.9% saline. Immediately the brains were dissected and the neurochemicals were estimated. ST, SN, hippocampus, cortex and cerebellum were dissected, immediately frozen on dry ice and stored at -80°C for western blot studies.

### Analysis of dopamine and serotonin

Dopamine and serotonin levels were measured in each supernatant by HPLC with electrochemical detection (Waters, Bangalore, India). Samples were injected using a Rheodyne 7725i injector valve with a 20 μL injection loop. The mobile phase consisting of 7% acetonitrile, 3% methanoland 90% 20 mM citric acid, 10 mM monobasic phosphate sodium, 3.25 mM octanesulfonic acid, 3 mM heptanesulfonic acid, 0.1 mM EDTA, 2 mM KCl, 6 mL/L o-phosphoric acid and 2 mL/L diethylamine (pH 3) was pumped at 0.3 mL min^−1^ with a Gold 118 system (Beckman, Fullerton, CA). Signals were recorded and quantified with a Beckman Gold 118integrator. Amounts of dopamine and serotonin were calculated by comparing peak levels from the supernatant samples with those of externalstandards. Monoamine levels were calculated as nM/mg weight tissue.

### Immunohistochemical studies

Serially sectioned SN was fixed in the gelatine coated slides and were deparaffinized in xylene and rehydrated in a graded series of ethanol. Then the slides were boiled in citrate buffer (10 mM, pH 6.0) for 15 min for antigen retrieval. To remove the endogenous peroxidase activity, they were incubated with 0.3% hydrogen peroxide (H_2_O_2_) for 10 min at room temperature. Then the slides were placed in blocking buffer containing 5% bovine serum albumin (BSA) with 0.2% Triton X-100 in 0.01 M PBS (pH 7.2) for 30 min at 37°C. During each and every treatment, the slides were washed at least three times with 0.01 M PBS. Then the sections were incubated for 24 h with primary anti mouse tyrosine hydroxylase (1:500) in 5% BSA, 0.2% Triton X-100 and 0.02% sodium azide in TBS. After washing with BSA in TBS, the sections were incubated in anti-mouse IgG-HRP-conjugated secondary antibody (1:1000) in BSA for one hour. Sections were washed with PBS and exposed to diaminobenzidine until the development of the colour. TH positive neurons in the SN were counted and boundary between the SN and ventral tegmental area was defined withthe aid of the mouse brain atlas [20]. The number of TH immunoreactive cells of the SN region by persons who were blind to the treatment. Cell counts were determinedevery sixth section (total 8–10 sections) through SN corresponding to the Bregma 2.92 mm to 3.64 mm from each of the animals, and three animals/group were used for cell counts. All rawcell counts were adjusted with a correction formula for cell sizeand section thickness according to the method of Abercrombie [21]. The cell counts werethen averaged for each animal and these averages were usedto calculate a mean ± SD for each treatment group.

RETRACTED

### Western blotting

Tissue samples were homogenized in RIPA buffer and centrifuged at 10,000 rpm for 30 min to isolate the supernatant. Protein amount was estimated according to method of Lowry et al. [22] and 50μg protein was loaded onto the polyacrylamide gels. Separated proteins were transferred onto PVDF membranes that were incubated overnight in the primary antibody for TH and α-synuclein (1:1,000, Cell Signalling, USA), DAT and VMAT 2 (1:1,000, Santa Cruz, USA) and β-actin (1:1,000, Sigma-Aldrich, USA). Membranes were washed with TBST and incubated with respective secondary antibodies conjugated with Horse reddish peroxidase (1:1,000) for 2 h. Protein bands were visualized by enhanced chemiluminescence method using ECL-kit (GenScript ECL kit, USA).

#### Image acquisition and densitometric analysis

In the present study, Total Lab 1.11 software version was used for image acquisition and densitometric analysis of the blots. It interpreted the raw data in three dimensions and the density was calculated as the total volume by forming two dimensions peak. It also contains tool to adjust the precise width of the band to account for the area under the shaded peak of interest. Then the blot intensities were compared their control values, which set as ‘100’.

### Data analysis

All data were expressed as mean ± Standard Deviation (SD) of number of experiments. The statistical significance was evaluated by one-way analysis of variance (ANOVA) using SPSS version 15.0 (SPSS, Cary, NC, USA) and the individual comparisons were obtained by Duncan’s Multiple Range Test (DMRT). A value of *P*< 0.05 was considered to indicate a significant difference between groups. Values sharing a common alphabet do not differ significantly with each other at *P*< 0.05.

## Results

### CMS exposure further enhances MPTP/p induced depletion of dopamine and serotonin

In PD, severe cognitive decline and mood alterations were found even prior to the occurrence of the motor symptoms. The nigrostriatal degeneration is responsible for the occurrence of motor features of PD, while extra-nigral degeneration corroborates to other non-motor symptoms, which are unresponsive to the gold standard drug L-DOPA. So, in order to investigate the initiative, progressive or concomitant role of the stressors on MPTP/p induced neurotoxicity in both nigral and extra-nigral regions, we sought to determine the levels of dopamine in striatum, cortex and hippocampus. HPLC- ECD analysis indicated that the levels of dopamine were high in the cortex and striatum as compared to the hippocampus in control mice. MPTP/p alone treatment and CMS alone exposure to mice significantly decreased dopamine levels in the studied brain regions. Exposure of stress or MPTP/p alone treatment induced less dopamine depletion as compared to pre and/or post stressed MPTP/p mice, which indicated the relationship between stress and pathological processes of PD. Post exposure of stress to MPTP/p treated animals induced more reduction in level of dopamine as compared to pre and pre&post stress exposed MPTP/p group, which also indicated that further neurodegeneration is induced by stress exposure (Fig 2).

RETRACTED

**Fig 2:** Effect of stress on the levels of dopamine in control and MPTP/p treated mice. The levels of dopamine in striatum, cortex and hippocampus were determined by HPLC- electrochemical method. Values are given as mean ± SD for six mice in each group. Values not sharing common alphabet differed significantly (P< 0.05) with each other.

In PD patients, the serotonin levels have been found to be diminished and serotonin enhancing drugs are generally used to treat PD associated depression. In both MPTP/p alone treated and CMS alone exposed mice showed significantly decreased serotonin levels in the striatum, cortex and hippocampus. Similar to dopamine levels, most reduction in the levels of serotonin were observed in the post stress exposed MPTP/p treated animals (Fig 3). The results of our present study indicated the diminished interaction between these two neurotransmitter systems in both nigral and extra-nigral tissues may contributed to PD-associated motor and non-motor symptoms.

**Fig 3:** Impact of stress on the levels of serotonin in control and MPTP/p treated mice. The levels of serotonin in nigrostriatal (A) and extra-nigrostriatal (B) were determined by HPLC- electrochemical method. Values are given as mean ± SD for six mice in each group. Values not sharing common alphabet differed significantly (P< 0.05) with each other.

### CMS further amplifies MPTP/p induced degeneration of TH immunopositive neurons

TH immunohistochemistry was performed to assess the survival of dopaminergic neurons in the control and experimental mice (Fig 4). In control mice, dopamine containing SN neurons were densely stained, whereas MPTP/p treated mice exhibited a marked loss of nigral dopaminergic neurons. Exposure to CMS also resulted in the slight depletion of TH-positive cells as compared to the control group, suggesting stress could damage dopaminergic neurons. Severe reduction of nigral TH immunoreactivity was observed in the chronic MPTP/p injected mice [23], whereas exposure to chronic restraint stress, oral treatment with corticosterone and concomitant CMS exposure [9,10]in rats did not alter the TH immunoreactivity as that of dopaminergic neurotoxin. But these stressors could exaggerate the loss of nigral TH cells in 6-OHDA treated rats, which is in line with our results. In addition to their combined known neurodamaging effects in the nigral tissue, stress and neurotoxin exposure has beenshown to exert theirdeleterious effect in extra-nigral neurons, which is a new finding.

RETRACTED

**Fig 4:** Effect of stress on immunoreactivity of TH positive cells in control and MPTP/p treated mice. Immunoreactivity of TH positive cells (A) in SN and quantified data (B) were shown. Values are given as mean ± SD for three mice in each group. Values not sharing common alphabet differed significantly (P< 0.05) with each other.

### CMS further depletes MPTP/p reduced TH, DAT and VMAT 2 expressions

TH is the rate limiting enzyme of the dopamine biosynthesis. The transport of dopamine is mediated by two transporters: DAT involved in the uptake of dopamine into neurons and VMAT 2 involved in the transport of monoamines including dopamine from neuronal cytosol into synaptic vesicles. Both of them played vital role in PD and their expressions have been altered in MPTP/p treated animals [24]. Till now, no studies showed the link between effects of stressors and expression of these two transporters proteins. Our results showed that TH, DAT and VMAT 2 were prominently expressed in the ST and midbrain of mice (Figs 5, 6 and 7), while equal expressions of TH but not DAT and VMAT 2 were found in the cortex, hippocampus and cerebellum (Figs 8, 9 and 10). MPTP/p treatment significantly decreased TH, DAT and VMAT 2 expressions in the ST and midbrain, but less significantly hippocampus, cortex and cerebellum of the C57BL/6 mice. Exposure to CMS alone affected TH, DAT and VMAT 2 protein expressions in all the studied brain regions examined with prominent reduction in frontal cortex. Post exposure of stress to PD animals induced more reduction in TH, DAT and VMAT 2 expressions as compared to pre and pre&post stress exposed MPTP/p group, which indicated that the post exposure of stress not only affected the biosynthesis, but also the transport of dopamine.

RETRACTED

**Fig 5:** Effect of stress on protein expression of TH in striatum and SN of control and -MPTP/p treated mice. Protein expression of TH (A) and quantified data (B) by densitometric analysis were shown. Values are expressed as arbitrary units and given as mean ± SD of three animals in each group. Values not sharing common alphabet differed significantly (P< 0.05) with each other.

**Fig 6:** Impact of stress on protein expression of DAT in striatum and SN of control and -MPTP/p treated mice. Protein expression of DAT (A) and quantified data (B) by densitometric analysis were shown. Values are expressed as arbitrary units and given as mean ± SD of three animals in each group. Values not sharing common alphabet differed significantly (P< 0.05) with each other.

**Fig 7:** Influence of stress on protein expression of VMAT 2 in striatum and SN of control and -MPTP/p treated mice. Protein expression of VMAT 2 (A) and quantified data (B) by densitometric analysis were shown. Values are expressed as arbitrary units and given as mean ± SD of three animals in each group. Values not sharing common alphabet differed significantly (P< 0.05) with each other.

**Fig 8:** Impact of stress on protein expression of TH in cortex, hippocampus and cerebellum of control and -MPTP/p treated mice. Protein expression of TH (A) and quantified data (B) by densitometric analysis were shown. Values are expressed as arbitrary units and given as mean ± SD of three animals in each group. Values not sharing common alphabet differed significantly (P< 0.05) with each other.

**Fig 9:** Influence of stress on protein expression of DAT in cortex, hippocampus and cerebellum of control and MPTP/p treated mice. Protein expression of DAT (A) and quantified data (B) by densitometric analysis were shown. Values are expressed as arbitrary units and given as mean ± SD of three animals in each group. Values not sharing common alphabet differed significantly (P< 0.05) with each other.

**Fig 10:** Effect of stress on protein expression of VMAT 2 in cortex, hippocampus and cerebellum of control and MPTP/p treated mice. Protein expression of VMAT 2 (A) and quantified data (B) by densitometric analysis were shown. Values are expressed as arbitrary units and given as mean ± SD of three animals in each group. Values not sharing common alphabet differed significantly (P< 0.05) with each other.

### CMS further enhances MPTP/p upregulated α-synuclein expression

The protein expression studies of α-synuclein (which plays a vital role in the pathogenesis and progression of PD) were performed in various brain regions of control and experimental mice. Protein expression studies showed the expression of α-synuclein was predominant in all the studied regions of brain (Figs 11 and 12). MPTP/p significantly enhanced the α-synuclein expression in the striatum and midbrain, but not in the hippocampus, cortex and cerebellum regions. CMS itself did not influence the expression of α-synuclein in all the studied brain regions, whereas post exposure of CMS exaggerates the expression of α-synuclein in MPTP/p treated mice.

RETRACTED

**Fig 11:** Effect of stress on protein expression of α-synuclein in striatum and SN of control and MPTP/p treated mice. Protein expression of α-synuclein (A) and quantified data (B) by densitometric analysis were shown. Values are expressed as arbitrary units and given as mean ± SD of three animals in each group. Values not sharing common alphabet differed significantly (P< 0.05) with each other.

**Fig 12:** Effect of stress on protein expression of α-synuclein in cortex, hippocampus and cerebellum of control and MPTP/p treated mice. Protein expression of α-synuclein (A) and quantified data (B) by densitometric analysis were shown. Values are expressed as arbitrary units and given as mean ± SD of three animals in each group. Values not sharing common alphabet differed significantly (P< 0.05) with each other.

### CMS facilitates MPTP/p induced motor impairments and anhedonia

To evaluate the motor disability and depression, various behavioural studies including open field, narrow beam walking and sucrose intake test were performed. Not surprisingly, MPTP/p group exhibited a significant decrease in movement (peripheral and central) and activities (rearing and grooming) in open field test (Fig 13) and time taken to cross the beam with enhanced foot slip errors showing motor impairments (Fig 14) and less pleasure to drink sweet water in sucrose intake test showing depression (Fig 15). Stress exposure similarly decreased the locomotion and activity and anhedonia in the mice. Separate exposure of stress or treatment with MPTP/p did not showsignificant change in motor and non-motor symptoms as compared to pre and/or post stressed MPTP/p mice.As similar to other parameters, we found that post exposure of stress to MPTP/p treated animals, to induce more changes in behaviour as compared to pre and pre&post stress exposed group.

**Fig 13:** Effect of stress on open field behavior of control and MPTP/p treated mice. The locomotion (peripheral (A) and central (B) movements) and activities (C) (grooming and rearing) were shown. Values are given as mean ± SD for six mice in each group. Values not sharing common alphabet differed significantly (P< 0.05) with each other.

**Fig 14:** Effect of stress on narrow beam walking test of control and MPTP/p treated mice. Time taken to cross the wooden beam (A) and number of foot slip errors (B) in narrow beam walking test were shown. Values are given as mean ± SD for six mice in each group. Values not sharing common alphabet differed significantly (P< 0.05) with each other.

RETRACTED

**Fig 15:** Effect of stress on sucrose intake levels in control and MPTP/p treated mice. The level of sucrose intake was shown. Values are given as mean ± SD for six mice in each group. Values not sharing common alphabet differed significantly (P< 0.05) with each other.

## Discussion

Previous studies indicated that the MPTP/p injection caused severe motor deficits, depletion of dopamine, loss of TH positive cells and reduced DAT and VMAT 2 expressions and enhanced α-synuclein expression in striatum and substantia nigra but not much severely in extra-nigral tissues. In addition, other studies reported that the stress exposure enhanced anhedonia and depletion of serotonin in extra-nigral tissues as compared to substantia nigra and striatum. Few experiments also indicated that the exposure of stress to 6-OHDA infused animals boost up the motor symptoms, dopamine depletion and loss of dopaminergic neurons. But none of the studies deals with the role of stressors on the non-motor symptoms, levels of monoamine, expression of dopaminergic markers and α-synuclein in extra-nigral tissues. Here we confirmed that post exposure of stress to MPTP/p treated mice worsened motor and non-motor symptoms by further augmenting monoamine depletion, degeneration of TH cells, decreased expression of DAT and VMAT 2 and increased expression of α-synuclein in both nigral and extra-nigral tissues.

Depression is considered as the most common non-motor symptom encountered by PD patients [25]. The etiology of depression in PD is complex, which may result from reduced brain levels of serotonin that is related with the central dopaminergic deficiency associated with PD motor symptoms [26,27]. Reduction in the levels of brain monoamines (dopamine and serotonin) in MPTP [28] and CMS [29] exposed mice were reported. Luchtman et al. [30,31] reported the differences in region specific depletion of dopamine in striatum, frontal cortex, midbrain, hippocampus and cortex in the chronic MPTP/p treated animals. Exposure to CMS also decreased the levels of dopamine and its metabolites in the striatum and cortex indicating an increased conversion of dopamine to its metabolites [32]. However, pre and/or post stress exposed MPTP/p treated mice showed a significant reduction in dopamine levels of all studied regions of brain as compared to PD or stress alone exposed mice. This indicates the relationship between PD and stress induced depression. Post exposure of stress to MPTP/p treated animals induced more reduction in dopamine levels as compared to pre and pre&post stress exposed MPTP/p group. Few unaffected dopaminergic neurons continue to synthesize and release dopamine after 6-OHDA lesion and this response become inadequate under chronic stress [33,34], which further support our present results and hypothesis.

RETRACTED

Studies have shown that serotonin neurons modulate dopamine function in all of the major dopamine pathways through a variety ofserotonin receptor subtypes that are differentially localized in dopamine-rich brain regions [35]. In our study, chronic administration of MPTP/p was associated with enhanced loss of serotonin in cortex and striatum as compared to other studied areas of brain. The central serotonergic system originates in the raphe nuclei and projects predominantly to cortical areas and the striatum [36]. PD is not only characterized by striatal dopaminergic terminal loss but also by serotonergic degeneration [37,38]. Vriend et al. [39] suggested that depression in PD arise mainly due to the hypo-dopaminergic state in the striatum. This may result in a lower stimulation of cortical brain areas that are associated with motivation and reward processing.

In our study, CMS appears to impair the serotonergic neurotransmission within the cortex and hippocampus as compared to other regions. Hippocampus, a key target of stress hormones, is predominantly connected with the prefrontal cortex, a region highly sensitive to environmental stimulation stress [40]. PD patients with depression symptoms have decreased cerebrospinal fluid concentrations of 5-hydroxyindol acetic acid, a serotonin metabolite, and reduced cortical 5-HT 1A receptor binding compared with PD patients not having depressive symptoms. On the one hand there are groups stating that serotonin exerts an inhibitory effect on striatal dopamine [41,42,43] and the reduced serotonin levels are often associated with a risk for depression [44]. On the other hand there are groups that have presented data stating that serotonin actually facilitates dopamine outflow [45,46]. This hypothesis considers a serotonin-induced dopamine release in the nucleus accumbens which is down-regulated by serotonin 2C receptors [47]. As a result, reductions in the serotonin content or increases in the serotonin 2C receptors inhibitory activity might be associated to the decline in dopaminergic neurotransmission in PD patients and subsequent worsening of mood symptoms. As like dopamine, pre and/or post stress exposed MPTP/p treated mice showed a significant reduction in serotonin levels of all studied regions of brain as compared to PD or stress alone exposed mice. Post exposure of stress to MPTP/p treated animals induced more reduction in serotonin levels as compared to pre and pre&post stress exposed MPTP/p group.

RETRACTED

Apart from dopamine, specific markers for PD such as TH, DAT and VMAT 2 [48,49], are involved in the biosynthesis and transport of dopamine. Chronic MPTP/p injection could induce a massive loss of dopaminergic neurons mainly in the SN as compared to a moderate loss in ventral tegmental area (VTA) [50]. Severe diminished expressions of these markers in striatum and SN [24] of chronic MPTP/p injected animals of the present study may result from the rapid death ofnigraldopaminergic neurons following the exposure to MPP^+^ [23,51]. Moderate decrease in the expression of dopaminergic markers in cortex, hippocampus and cerebellum of MPTP/p injected mice might be due to the moderate dopamine cell loss in VTA [52,53]. Rasheed et al. [54] reported that down regulation of TH expression occurs during CMS exposure in various brain regions, which is also consistent with our study. The reduced dopamine levels during CMS exposure may reduce the DAT expression slightly [55]. The chronic stress decreased density of VMAT 2 and may result in preferential monoamine accumulation in the cytoplasm as a consequence of reduced vesicular storage capability [56]. In post-mortem studies, a decrease in dopamine neurons in the VTA was detected in depressed PD patients [57]. Pre and/or post stress exposed MPTP/p treated mice showed significant reduction in the expressions of TH, DAT and VMAT 2 as compared to PD or stress alone exposed mice indicated that the stress is responsible for further disruption of dopaminergic neurons associated with PD.

A histological hallmark of PD is the presence of fibrillar aggregates called Lewy bodies (LBs), in which α-synuclein is a major constituent. α -synuclein counter-act a toxic injury and its expression could affect specific stress signalling pathways linked to neuronal survival [58]. Significant enhanced expression of α-synuclein found in striatum and SN of MPTP/p treated mice can confer protection against MPTP-induced neurodegeneration. Its expression is enhanced less significantly in other regions of brain including hippocampus; cortex and cerebellum may be due to moderate cell loss in VTA. Lewy body deposition in brainstem areas implicated in depression, including the serotoninergic raphe nuclei and the noradrenergic locus coeruleus [59,60], can precede basal midbrain involvement in PD [61]. This may explain theoccurrence of depression and anxiety in PD during the premotor phase [62]. However exposure to CMS did not alter the expressions of α-synuclein in all the above studied brain regions, which clearly indicates the difference in pathogenesis of major depression compared to PD with depressive symptoms.

RETRACTED

Open field test is normally used to assess locomotor, exploratory and anxiety-like behaviour in experimental rodents (rats/mice). Reduced performance of MPTP/p animals in crossing peripheral and central squares and activities (grooming and rearing) may be due to reduced dopaminergic loss in SN [63]. In the open field test, CMS mice exhibited decreased acclimatization and exploratory behaviour with enhanced grooming and rearing activities. Decreased mobility and enhanced grooming activity depicts a higher level of anxiety [64]. Moreover decreased motor activity as a consequence of severe stress has been widely reported, as indicator for ‘depressive-like’ behaviour [65]. Exposure of pre or/and post stress to MPTP/p animals showed more reduction in movement and enhancement in grooming activities, indicated more dopaminergic loss and anxiety in these animals as compared to MPTP/p or stress alone exposed animals.

The narrow beam walking test was used to test the balance, vestibular integrity and muscular co-ordination [63,66]. In narrow beam walking, the MPTP animals showed more deficits in crossing time with enhanced foot slip errors as compared to stress alone exposed animals. Exposure of pre or/and post stress to MPTP/p animals showed more time taken to cross the beam with more slip error indicated more dopaminergic loss in these animals as compared to MPTP/p or stress alone exposed animals.

Sucrose intake test is used to measure anhedonia, a decreased ability to experience pleasure, is a core symptom of human depression [67]. However, in this study, chronic MPTP/p injection did not induce anhedonia. CMS and pre or/and post CMS exposure to MPTP/p mice depressed the consumption and preference for, palatable, sweet solutions as indicated by Willner et al. [18]. DA neuronal functioning is fundamental in sub serving reward processes [68], although other neurotransmitters (e.g. serotonin) like wise contribute in this respect [69]. Response for rewarding can be elicited from a number of dopamine rich areas, as well as regions containing fibers of passage. Specifically, dopamine activity is altered within the cortex and nucleus accumbens, but nigrostriatal dopamine functioning seems less affected by stressors [70,71].

The present study demonstrates that chronic stress exposure following neurotoxin-induced neurodegeneration exacerbates the behavioural dysfunction and degeneration of the nigrostriatal/non-nigrostriatal dopaminergic systems rather than concurrent with or preceding ones. Depression in PD is not merely considered as secondary to the psychological stress of a chronic disease itself and associated disability but it could be a result from neuroanatomical changes that occurred due to neurodegeneration [72]. Our study clearly indicated that the anhedonia is mainly occurred due to the loss of monoamines and its related markers. Results of the present study indicate that the stress accelerated pathological changes in PD and suggests a new therapeutic path for using drugs that treat mood and motor aspects of this disorder during the course of the disease.

RETRACTED

## Supporting Information

S1 Dataset The data set and supporting information for Figs 2, 3 and 4. (XLSX)

S2 Dataset The data set and supporting information for Figs 5, 6 and 7. (XLSX)

S3 Dataset The data set and supporting information for Figs 8, 9 and 10. (XLSX)

S4 Dataset The data set and supporting information for Figs 11 and 12. (XLSX)

S5 Dataset The data set and supporting information for Figs 13, 14 and 15. (XLSX)

## References

[1] HornykiewiczO (1975) Brain monoamines and parkinsonism. Natl Inst Drug Abuse Res Monogr Ser 3: 13–21. 78779610.1037/e472122004-001

[2] UcEY, TippinJ, ChouKL, EricksonBA, DoerschugKC, Jimmeh FletcherDM (2012) Non-motor Symptoms in Parkinson’s Disease. European Neurological Review 7: 35–40. 10.17925/ENR.2012.07.01.35

[3] ModugnoN, LenaF, DibiasioF, CerroneG, RuggieriS, FornaiF (2013) A clinical overview of non-motor symptoms in Parkinson’s disease. Archives Italiennes de Biologie 151: 148–168. 24873924

[4] SwaabDF, BaoAM, LucassenPJ (2005) The stress system in the human brain in depression and neurodegeneration. Ageing Res Rev 4: 141–194. 1599653310.1016/j.arr.2005.03.003

[5] AarslandD, MarshL, SchragA (2009) Neuropsychiatric symptoms in Parkinson's disease. Mov Disord 24: 2175–2186. 10.1002/mds.22589 19768724PMC2787875

[6] GoetzCG, TannerCM, PennRD, StebbinsGT, GilleyDW, ShannonKM et al (1990) Adrenal medullary transplant to the striatum of patients with advanced Parkinson’s disease: 1-year motor and psychomotor data. Neurology 40: 273–276. 230024810.1212/wnl.40.2.273

[7] TrevesTA, RabeyJM, KorczynAD (1990) Case-control study, with use of temporal approach, for evaluation of risk factors for Parkinson’s disease. Movement Dis 5: 11.

[8] SmithAD, CastroSL, ZigmondMJ (2002) Stress-induced Parkinson’s disease: a working hypothesis. Physiol Behav 77: 527–531. 1252699410.1016/s0031-9384(02)00939-3

[9] SmithLK, JadavjiNM, ColwellKL, Katrina PerehudoffS, MetzGA (2008) Stress accelerates neural degeneration and exaggerates motor symptoms in a rat model of Parkinson's disease. Eur J Neurosci 27: 2133–2146. 10.1111/j.1460-9568.2008.06177.x 18412632PMC5222623

RETRACTED

[10] HemmerleAM, DickersonJW, HermanJP, SeroogyKB (2014) Stress exacerbates experimental Parkinson’s disease. Mol Psychiatry 19: 638–640. 10.1038/mp.2013.108 23999522

[11] MonroeSM, TorresLD, GuillaumotJ, HarknessKL, RobertsJE, FrankE et al (2006) Life stress and the long-term treatment course of recurrent depression: Non severe life events predict recurrence for medicated patients over 3 years. J Consult Clin Psychol 74: 112–120. 1655114810.1037/0022-006X.74.1.112

[12] WillnerP (2005) Chronic mild stress (CMS) revisited: consistency and behavioural-neurobiological concordance in the effects of CMS. Neuropsychobiology 52: 90–110. 1603767810.1159/000087097

[13] SchragA (2006) Quality of life and depression in Parkinson's disease. J Neurol Sci 248: 151–157. 1679702810.1016/j.jns.2006.05.030

[14] McEwenBS (2005) Glucocorticoids, depression, and mood disorders: structural remodeling in the brain. Metabolism 54: 20–23. 1587730810.1016/j.metabol.2005.01.008

[15] PacakK, PalkovitsM (2001) Stressor specificity of central neuroendocrine responses: implications for stress-related disorders. Endocr Rev 22: 502–548. 1149358110.1210/edrv.22.4.0436

[16] AlaladeE, DennyK, PotterG, SteffensD, WangL (2011) Altered cerebellar-cerebral functional connectivity in geriatric depression. PLoS ONE.6: e20035 10.1371/journal.pone.0020035 21637831PMC3102667

[17] PetroskeE, MeredithGE, CallenS, TotterdellS, LauYS (2001) Mouse model of parkinsonism: a comparison between Subacute MPTP and chronic MPTP/probenecid treatment. Neurosci 106: pp. 589–601.10.1016/s0306-4522(01)00295-011591459

[18] WillnerP, TowellA, SampsonD, SophokclousS, MuscatR (1987) Reduction of sucrose preference by chronic unpredictable mild stress, and its restoration by a tricyclic antidepressant. Psychopharmacology (Berl) 93: 358–64. 312416510.1007/BF00187257

[19] RajaSankarS, ManivasagamT, SurendranS (2009) Ashwagandha leaf extract: a potential agent in treatingoxidative damage and physiological abnormalities seen in amouse model of Parkinson's disease. Neurosci Lett 454: 11–15. 10.1016/j.neulet.2009.02.044 19429045

[20] LowryOH, RosebroughNJ, FarrAL, RandallRJ (1951) Protein measurement with the Folin phenol reagent. J Biol Chem 193: 265–275. 14907713

[21] FranklinKBJ, PaxinosG (2007) The mouse brain in stereotaxic coordinates. London: Academic Press.

[22] AbercrombieM (1946) Estimation of nuclear population from microtome sections. Anat Rec 94:239–247. 2101560810.1002/ar.1090940210

[23] NicklasWJ, YoungsterSK, KindtMV (1987) MPTP, MPP^+^ and mitochondrial function. Life Sci 40: 721–729. 310089910.1016/0024-3205(87)90299-2

[24] AnandhanA, TamilselvamK, RadhigaT, RaoS, EssaMM, ManivasagamT (2012) Theaflavin, a black tea polyphenol, protects nigral dopaminergic neurons against chronic MPTP/probenecid induced Parkinson's disease. Brain Res 1433: 104–113. 10.1016/j.brainres.2011.11.021 22138428

RETRACTED

[25] LohleM, StorchA, ReichmannH (2009) Beyond tremor and rigidity: non-motor features of Parkinson's disease. J Neural Transm 116: 1483–1492. 10.1007/s00702-009-0274-1 19680598

[26] MayeuxR (1990) Depression in the patient with Parkinson's disease. J Clin Psychiatry 51: 24–5. 2195009

[27] MayeuxR, WilliamsJB, SternY, CoteL (1984) Depression and Parkinson's disease. Adv Neurol 40: 241–50.6695601

[28] PainS, GochardA, BodardS, GulhanZ, Prunier-AeschC, ChalonS (2013) Toxicity of MPTP on neurotransmission in three mouse models of Parkinson's disease. Exp Toxicol Pathol 65: 689–94. 10.1016/j.etp.2012.09.001 23083629

[29] VancasselS, LemanS, HanonickL, DenisS, RogerJ, NolletM et al (2008) n−3 polyunsaturated fatty acid supplementation reverses stressinduced modifications on brain monoamine levels in mice. J Lipid Res 49: 340–348. 1799175710.1194/jlr.M700328-JLR200

[30] LuchtmanDW, ShaoD, SongC (2009) Behavior, neurotransmitters and inflammation in three regimens of the MPTP mouse model of Parkinson's disease. Physiol Behav 98: 130–138. 10.1016/j.physbeh.2009.04.021 19410592

[31] LuchtmanDW, MengQ, SongC (2012) Ethyl-eicosapentaenoate (E-EPA) attenuates motor impairments and inflammation in the MPTP-probenecid mouse model of Parkinson’s disease. Behav Brain Res 226: 386–396. 10.1016/j.bbr.2011.09.033 21971013

[32] JavelotH, MessaoudiM, JacquelinC, BissonJF, RozanP, NejdiA et al (2014) Behavioral and neurochemical effects of dietary methyl donor deficiency combined with unpredictable chronic mild stress in rats. Behav Brain Res 261: 8–16. 10.1016/j.bbr.2013.11.047 24333542

[33] AbercrombieED, KeefeKA, DiFrischiaDF, ZigmondMJ (1989) Differential effects of stress on *in vivo* dopamine release in striatum, nucleus accumbens, and medial frontal cortex. J Neurochem 52: 1655–1658. 270901710.1111/j.1471-4159.1989.tb09224.x

[34] KeefeKA, StrickerEM, ZigmondMJ, AbercrombieED (1990) Environmental stress increases extracellular dopamine in striatum of 6-hydroxydopamine-treated rats: in vivo micro dialysis studies. Brain Res 527: 350–353. 212373010.1016/0006-8993(90)91158-d

[35] AlexKD, PehekEA (2007) Pharmacologic mechanisms of serotonergic regulation of dopamine neurotransmission. Pharmacol Ther 113: 296–320. 1704961110.1016/j.pharmthera.2006.08.004PMC2562467

[36] MichelsenKA, PrickaertsJ, SteinbuschHW (2008) The dorsal raphe nucleus and serotonin: implications for neuroplasticity linked to major depression and Alzheimer’s disease. Prog Brain Res 172: 233–246. 10.1016/S0079-6123(08)00912-6 18772036

RETRACTED

[37] KishSJ, TongJ, HornykiewiczO, RajputA, ChangLJ, GuttmanM et al (2008) Preferential loss of serotonin markers in caudate versus putamen in Parkinson’s disease. Brain 131: 120–131. 1795690910.1093/brain/awm239

[38] HirschEC, OrieuxG, MurielMP, FrancoisC, FegerJ (2003) Nondopaminergic neurons in Parkinson’s disease. Adv Neurol 91: 29–37. 12449099

[39] VriendC, PattijT, van der WerfYD, VoornP, BooijJ, RuttenS et al (2013) Depression and impulse control disorders in Parkinson's disease: two sides of the same coin? Neurosci Biobehav Rev 38C: 60–71. 10.1016/j.neubiorev.2013.11.001 24239733

[40] JayTM, RocherC, HotteM, NaudonL, GurdenH, SpeddingM (2004) Plasticity at hippocampal to prefrontal cortex synapses is impaired by loss of dopamine and stress: Importance for Psychiatric diseases. Neurotox Res 6: pp. 233–244. 1532596210.1007/BF03033225

[41] De DeurwaerdereP, NavaillesS, BergKA, ClarkeWP, SpampinatoU (2004) Constitutive activity of the serotonin2C receptor inhibits in vivo dopamine release in the rat striatum and nucleus accumbens. J Neurosci 24: 3235–3241. 1505670210.1523/JNEUROSCI.0112-04.2004PMC6730027

[42] Di MatteoV, CacchioM, Di GiulioC, EspositoE (2002) Role of serotonin (2C) receptors in the control of brain dopaminergic function. Pharmacol Biochem Behav 71: 727–734. 1188856410.1016/s0091-3057(01)00705-5

[43] JacobsBL, FornalCA (1993) 5-HT and motor control: a hypothesis. Trends Neurosci 16: 346–352. 769440310.1016/0166-2236(93)90090-9

[44] Van PraagHM, De HaanS (1979) Central serotonin metabolism and frequency of depression. Psychiatry Res 1: 219–224. 9523310.1016/0165-1781(79)90002-7

[45] BenloucifS, GallowayMP (1991) Facilitation of dopamine release in vivo by serotonin agonists: studies with microdialysis. Eur J Pharmacol 200: 1–8. 176936610.1016/0014-2999(91)90658-d

[46] BenloucifS, KeeganMJ, GallowayMP (1993) Serotonin-facilitated dopamine release in vivo: pharmacological characterization. J Pharmacol Exp Ther 265: 373–377. 8474019

[47] DremencovE, NewmanME, KinorN, Blatman-JanG, SchindlerCJ, OverstreetDH et al (2005) Hyperfunctionality of serotonin-2C receptor-mediated inhibition of accumbal dopamine release in an animal model of depression is reversed by antidepressant treatment. Neuropharmacology 48: 34–42. 1561772510.1016/j.neuropharm.2004.09.013

[48] HeikkilaRE, SonsallaP (1992) The MPTP-treated mouse as a model of parkinsonism: How good is it. Neurochem Int 20: 299–303. 136544610.1016/0197-0186(92)90256-q

[49] MillerGW, EricksonJD, PerezJT, PenlSN, MashDC, RyeDB et al (1999) Immunochemical analysis of vesicular monoamine transporter (VMAT2) protein in Parkinson’s disease. Exp Neurol 156: 138–148. 1019278510.1006/exnr.1998.7008

RETRACTED

[50] AhmadSO, ParkJH, BittelLS, LauYS (2009) Effects of endurance exercise on ventral tegmental area neurons in the chronic 1-methyl-4-phenyl-1,2,3,6-tetrahydropyridine and probenecid-treated mice. Neurosci Lett 450: 102–105. 10.1016/j.neulet.2008.11.065 19084578

[51] DawsonTM (2000) New animal models for Parkinson’s disease. Cell 101: 115–118. 1078683010.1016/S0092-8674(00)80629-7

[52] LiuB, XieJX, RowlandsDK, GouYL, LeungCC, ChungYW et al (2004) Neuroprotective effects of Bak Foong Pill in 1-methyl-4-phenyl-1,2,3,6-tetrahyrdropyridine (MPTP)-induced Parkinson's disease model mice. Biol Pharm Bull 27: 1245–50. 1530503010.1248/bpb.27.1245

[53] LismanJE, GraceAA (2005) The hippocampal-VTA loop: controlling the entry of information into long-term memory. Neuron 46: 703–13. 1592485710.1016/j.neuron.2005.05.002

[54] RasheedN, AhmadA, Al-SheehaM, AlghashamA, PalitG (2011) Neuroprotective and anti-stress effect of A68930 in acute and chronic unpredictable stress model in rats. Neurosci Lett 504: 151–15. 10.1016/j.neulet.2011.09.021 21945949

[55] IkawaK, WatanabeA, KanenoS, ToruM (1993) Modulation of (³H)mazindol binding sites in rat straitum by dopaminergic agents. Eur J Pharmacol 250: 261–266. 790665310.1016/0014-2999(93)90390-4

[56] SchmitzY, LeeCJ, SchamaussC, GononF, SulzerD (2001) Amphetamine distorts stimulation-dependent dopamine overflow: effects on D2 auto receptors, transporters, and synaptic vesicle stores. J Neurosci 21: 5916–5924. 1148761410.1523/JNEUROSCI.21-16-05916.2001PMC6763160

[57] BrownAS, GershonS (1993) Dopamine and depression. J Neural Transm Gen Sect 91: 75–109. 809980110.1007/BF01245227

[58] HashimotoM, HsuLJ, SiskA, XiaY, TakedaA, SundsmoM et al (1998) Human recombinant NACP/alpha-synuclein is aggregated and fibrillated in vitro: relevance for Lewy body disease. Brain Res 799: 301–306. 967531910.1016/s0006-8993(98)00514-9

[59] ItoiK, SugimotoN (2010) The brainstem noradrenergic systems in stress, anxiety and depression. J Neuroendocrinol 22: 355–361. 10.1111/j.1365-2826.2010.01988.x 20210846

[60] LowryCA, HaleMW, EvansAK, HeerkensJ, StaubDR, GasserPJ et al (2008) Serotonergic systems, anxiety, and affective disorder: focus on the dorsomedial part of the dorsal raphe nucleus. Ann N Y Acad Sci 1148: 86–94. 10.1196/annals.1410.004 19120094

[61] BraakH, BohlJR, MüllerCM, RübU, de VosRA, Del TrediciK (2006) Stanley Fahn Lecture 2005: the staging procedure for the inclusion body pathology associated with sporadic Parkinson's disease reconsidered. Mov Disord 21: 2042–2051. 1707804310.1002/mds.21065

[62] ShibaM, BowerJH, MaraganoreDM, McDonnellSK, PetersonBJ, AhlskogJE et al (2000) Anxiety disorders and depressive disorders preceding Parkinson's disease: a case—control study. Mov Disord 15: 669–677. 1092857710.1002/1531-8257(200007)15:4<669::aid-mds1011>3.0.co;2-5

RETRACTED

[63] CrabbeJC, MettenP, Chia-HuaY, SchlumbohmJP, CameronAJ, WahlstenD (2003) Genotypic differences in ethanol sensitivity in two tests of motor in coordination. J Appl Physiol 95: 1338–1351. 1270409010.1152/japplphysiol.00132.2003

[64] BhattacharyaSK, BhattacharyaA, ChakrabartiA (2000) Adaptogenic activity of Siotone, a polyherbal Ayurvedic rasayana formulation. Indian J Exp Biol 38: 119–128. 11218827

[65] AnismanH, ZacharkoRM (1982) Depression: the predisposing influence of stress. Behav Brain Sci 5: 89–137. 10.1017/S0140525X00010633

[66] FlemingSM, SalcedoJ, FernagutP-O, RockensteinE, MasliahE, LevineMS et al (2004) Early and progressive sensorimotor anomalies in mice overexpressing wild-type human α-synuclein. J Neurosci 24: 9434–9440. 1549667910.1523/JNEUROSCI.3080-04.2004PMC6730110

[67] KesslerRC, McGonagleKA, ZhaoS, NelsonCB, HughesM, EshlemanS (1994) Lifetime and 12-month prevalence of DSM-III-R psychiatric disorders in the United States. Results from the National Comorbidity Survey. Arch Gen Psychiatry 51: 8–19. 827993310.1001/archpsyc.1994.03950010008002

[68] WiseRA (1985) The anhedonia hypothesis: mark III. Behav Brain Sci 8: 178–186.

[69] HarrisonAA, MarkouA (2001) Serotonergic manipulations both potentiate and reduce brain stimulation reward in rats: involvement of serotonin-1A receptors. J Pharmacol Exp Ther 297: 316–325. 11259559

[70] DeutchAY, BourdelaisAJ, ZahmDS (1993) The nucleus accumbens core and shell: accumbal compartments and their functional attributes In: KalivasP.W., BarnesC.D., (Eds.), Limbic Motor Circuits and Neuropsychiatry. CRC Press, Boca Raton, FL, pp. 45–88.

[71] DeutchAY, TamSY, RothRH (1985) Footshock and conditioned stress increase 3,4-dihydroxyphenylacetic acid (DOPAC) in the ventral tegmental area but not substantia nigra. Brain Res. 333, 143–146. 399528210.1016/0006-8993(85)90134-9

[72] McDonaldWM, RichardIH, DeLongMR (2003) Prevalence, etiology, and treatment of depression in Parkinson's disease. Biol Psychiatry 54: 363–375. 1289311110.1016/s0006-3223(03)00530-4

